# Environmental impact of submerged and emerged breakwaters

**DOI:** 10.1016/j.heliyon.2022.e12626

**Published:** 2022-12-23

**Authors:** Cherdvong Saengsupavanich, Effi Helmy Ariffin, Lee Shin Yun, Dunstan Anthony Pereira

**Affiliations:** a Faculty of International Maritime Studies, Kasetsart University, Sri Racha Campus, 199 Moo 6 Sukhumvit Rd., Tungsukla, Sri Racha, Chonburi, 20230, Thailand; b Institute of Oceanography and Environment, Universiti Malaysia Terengganu, 21030, Kuala Nerus, Terengganu, Malaysia; c Faculty of Science and Marine Environment, Universiti Malaysia Terengganu, 21030, Kuala Nerus, Terengganu, Malaysia; d Coastal Management & Oceanography Research Centre, National Water Research Institute of Malaysia, Ministry of Natural Resources, Environment and Climate Change, 43300, Seri Kembangan, Selangor, Malaysia

**Keywords:** Coastal erosion, Coastal protection structures, Hard options, Engineering solutions, Beach conservation

## Abstract

Coastlines are constantly threatened by erosion. Effective coastal defense structures with the least environmental impacts are increasingly required. Submerged and emerged breakwaters have been implemented globally, while positively or negatively creating impacts on the environment. One of the most significant concerns in applying breakwaters is how to minimize their undesirable consequences on the environment. Thus, a thorough understanding of how submerged and emerged breakwaters affect the surrounding environment must be achieved. This article critically reviews and summarizes their environmental impacts on beach morphology, hydrodynamics, ecology, tourism, and recreation, as well as other notable impacts. This is a review article that may help coastal practitioners to manage coastal erosion with breakwaters more sustainably.

## 1 Introduction

Coastal zones are highly productive and valued globally for their natural resources, which supply humans with a variety of crucial goods and services such as recreational opportunities and protection against flooding, and economic benefits from the tourism, shipping, and fishery industries (Mehvar et al., 2018; Ratnayake and Perera, 2022). They are susceptible to climate change (Mohd et al., 2018; Sharaan et al., 2022) because of their vulnerability when exposed to extreme events such as strong winds, storm surges, cyclones, floodings, and sea-level rise (Palamakumbure et al., 2020; Perera et al., 2022). At present, coastal zones are undergoing rapid population growth, land conversion, and urbanization (Gunasinghe et al., 2021; Petrişor et al., 2020; Strain et al., 2022). Nearly half of the global population currently lives within 200 km of the coast, and the projected statistics show that the population growth could reach 70% by 2025 (Bagheri et al., 2021). However, coastal erosion in most sea-connected countries is a threat that has not been completely solved (Saengsupavanich, 2020a; Sanitwong-Na-Ayutthaya et al., 2022; Setyawan, 2022; Uda, 2022). The erosion from either anthropogenic or natural causes critically harms coastal settlements, infrastructure, and the community’s well-being (Saengsupavanich, 2019, 2020b). Various coastal protection measures are available, including soft and hard measures. The soft solutions often involve non-structural techniques, such as beach nourishment (Pinto et al., 2020), vegetation cover (Gomez et al., 2020), and mangrove afforestation (Gijón Mancheño et al., 2021). On the other hand, the hard options are related to structures that do not develop naturally, such as rocks, concrete, steel, or timber (Siegel, 2020).

Breakwaters, both submerged and emerged, represent a common approach to shoreline defense and provide substantial protection against severe storm conditions, reducing risks to coastal communities and local economic activities (Mohamed Rashidi et al., 2021; Silva et al., 2017). In Thailand, it has been used to protect harbors and eroded coastlines (Prukpitikul et al., 2019). Uda (2022) showed that breakwaters were installed at many Japanese ports such as Oharai Port, and Fukude Fishing Port, as well as along Japan’s eroded shorelines such as Ichiki and Kushikino coasts. The application of breakwaters in Indonesia was proven successful in protecting the coast and rehabilitating mangrove forest (Akbar et al., 2017). In Malaysia, several emerged and submerged breakwaters were constructed to solve coastal erosion (Mohamed Rashidi et al., 2021). Similar applications to protect coastlines while promoting mangroves and marshes can be found in many countries (Martin et al., 2021). Although the effectiveness of breakwaters is well-realized, there have been numerous publications on their negative impacts. Betzold et al. (2017) argued that hard coastal structures artificially fix the coastline but compromise the ability of beaches to adapt to changing conditions, leading to passive and aggressive ecological consequences. Breakwaters also significantly interrupt nearshore hydrodynamic regimes and sediment transport (Amalan et al., 2018; Le Xuan et al., 2022), affecting surrounding assemblage structures (Martins et al., 2009). Some researchers consider breakwaters to be non-adaptive, as they are costly to build and to maintain in response to a changing climate (Schoonees et al., 2019).

Breakwaters can secure eroding coastlines and support economic, as well as social, activities (Saengsupavanich, 2013a), while positively or negatively inducing physical and ecological impacts on the coastal environment. One of the most significant concerns in applying breakwaters is how to minimize their undesirable consequences on the environment. Before minimizing such impacts, a thorough understanding of how submerged and emerged breakwaters affect the surrounding environment must be achieved. This article reviews their economic considerations and summarizes their impacts on beach morphology, hydrodynamics, ecology, coastal tourism, and recreation, and other notable effects. Coastal practitioners can utilize this article as a tool to sustainably apply breakwaters in coastal protection.

## 2 Submerged breakwaters

Submerged breakwaters are low-crested offshore structures that are built shore-parallel in shallow water, with their crests at or below water level. Submerged breakwaters cover vertical breakwaters, rubble mound breakwaters, semi-circular breakwaters, and geosynthetic breakwaters (Na’im et al., 2018; Young and Testik, 2011). They can be used to improve port maneuvering and control sedimentation by regulating water currents and creating wave-interference zones (Eryani, 2019). Their geometry (e.g., crest, front slope, and back slope) plays a significant role in determining their effectiveness. Lately, submerged breakwaters have become more prevalent than emerged breakwaters (Na’im et al., 2018). Since utilizing submerged breakwaters to prevent coastal erosion is more popular internationally, an issue has arisen whether they can protect beaches and enhance the environment (Sulaiman and Hidayat, 2020; Torres-Freyermuth et al., 2019; Zanuttigh, 2007). Whether the environmental impacts of submerged breakwaters are well-understood is a major remaining question. In this section, various publications are collected, reviewed, and highlighted under different categories of their impacts on the coastal environment.

### 2.1 Economic considerations

Recognizing the economic necessity of maintaining shorelines and beaches to protect the livelihood of local inhabitants, submerged breakwaters offer a potential economic solution. Their construction cost may be comparatively cheaper because of their relatively lower crest elevation, requiring less construction materials. When the crest height is lower, an overall structural weight is reduced, and piles may not be required. In Ostia, Italy, Tomasicchio and Member (1996) compared the submerged and emerged breakwaters and concluded that there was no cost difference between applying them. Cho et al. (2001) also advocated a trapezoidal-shaped submerged breakwater because it was more economical and had the smallest sectional area than other shapes. Narayan et al. (2016) conducted a cost analysis between engineering structures and nature-based defense projects and found that submerged breakwaters cost two to five times more than natural defenses like mangroves and salt marshes. Pranzini et al. (2018) and Sulaiman and Hidayat (2020) found that low-crested breakwaters were relatively economical and affordable to the community, and they expected to apply low-crested breakwaters to not only shallow beaches, but also more universally to deeper coastal waters with harsher wave conditions. Furthermore, the construction costs can differ in different circumstances. Zahra et al. (2018) estimated the economic losses caused by submerged breakwater construction delay and found that such delay could cost more than 30% of the original cost. Additionally, the construction cost of submerged breakwaters can vary greatly with each country. Hillen et al. (2010) found that the construction budget in Vietnam could be ten times less than that in the USA and in European countries because of the lower labor and material prices.

### 2.2 Impact on beach morphology

Although submerged breakwaters induce beach morphological changes under a combination of wave and current actions, such changes are less dramatic than those induced by emergent breakwaters. There is a discrepancy in the conclusion on how beaches behind submerged breakwaters are affected.

Sulaiman and Hidayat (2020) and Fitri et al. (2019) showed that submerged breakwaters significantly impacted beach realignment. Their results showed that there was a formation of salient and tombolo behind structures. Sedimentation pattern, shoreline, and bottom shape change in front of submerged breakwater were noticed by Zahra (2018). An integrated study of sedimentological and morphosedimentary was carried out by Pennetta (2018), who found an accretion on the updrift side of submerged breakwaters, while erosion was intensely marked on the downdrift side. Ranasinghe and Sato (2007) studied the performance of a submerged breakwater on a littoral drift and found that the downdrift zone of the submerged breakwater was subjected to erosion because of the deficit of the sediment supply, steepening the foreshore. This phenomenon further accelerated the erosion until beach morphology reached an equilibrium. Interestingly, when coastal equilibrium was attained, sand moving from updrift to downdrift promoted salient formation and reduced further erosion on the downdrift.

In addition to simultaneous updrift deposition and downdrift erosion created by submerged breakwaters, many researchers found different patterns of beach morphological adjustment. In Italy, the coastline at Senzuno changed from being a natural straight linear feature to a salient-bay shape by constructing an emerged, segmented breakwater system, then back to a more linear beachfront by modifying the emergent breakwaters to a submerged continuous structure (Pranzini et al., 2018). According to Kamali et al. (2010), who undertook a study on a combination of low-crested breakwaters and mangrove restoration in Malaysia, morphological sediment deposition was formed behind the low-crested breakwaters. Substrate elevation was increased to a height appropriate for mangrove establishment. Sulaiman and Hidayat (2020) also noticed an alteration in the coastline that seemed to be eroded at both ends of low-crested breakwaters. Torres-Freyermuth et al. (2019) presented a similar finding, identifying the role of low-crest detached breakwaters on the morphological response on the Mexico’s northern Yucatan coast. The flanking phenomenon occurred, whereby the diffraction process at both ends of low-crested breakwaters eroded the adjacent areas. On the other hand, a case study carried out by Kubowicz-Grajewska (2015) claimed that submerged breakwaters had no significant impact on modifying offshore and nearshore morphology. Their findings showed a clear conflict with other publications on the formation of salient and tombolo after implementing submerged breakwaters.

Scouring around submerged and emerged breakwaters has been extensively discussed (Fredsøe and Sumer, 1997; Garcia and Kobayashi, 2015; Lorenzoni et al., 2016; Sumer et al., 2005). A quite extensive review regarding the scour involving submerged breakwaters was presented by Sumer et al. (2001). Scour holes around breakwaters could eventually lead to deterioration and damage of the structures (Salauddin and Pearson, 2019). A few researchers mentioned that scouring could affect beach morphology, tidal patterns, local turbidity levels, and benthic communities in the vicinity of breakwaters (Heery et al., 2017; Mulvihill and Beeman, 1980; Toso et al., 2019).

### 2.3 Impact on hydrodynamics

Submerged breakwaters change the surrounding hydrodynamics such as waves and water current patterns. Submerged breakwaters significantly reduce incoming wave heights, forcing waves to break upon their crests (Martin et al., 2021; Vona et al., 2020). Rubble mound breakwaters can be constructed with low levels of crest, allowing wave overtopping during storms (Kamali et al., 2010). Wave energy is absorbed by rocks or concrete units on the armor layer, preventing gravel or sand from seeping out of the core of the breakwater. Submerged breakwaters protect eroding coastline, lowering upland migratory pressure and enabling natural marsh areas to grow. Martin et al. (2021) showed that fringing marsh in Alabama retreated upland dramatically without breakwater protection. Zahra (2018) concluded that submerged breakwaters were an ideal approach for protecting a bay in Egypt since they reduced wave impact while allowing wave passage, avoiding their adverse effects on adjacent areas. Additionally, a study by Pranzini et al. (2018) found that widening the crest of a submerged breakwater can reduce the risk of a scour trough forming on the landward side of the structure.

Water currents and related sedimentation are affected by submerged breakwaters. In Malaysia, Fitri et al. (2019) studied the hydrodynamic mechanism of low-crested detached breakwaters on a muddy coast. Wave overtopping induced a suspended sediment flow on the leeward side of the submerged breakwaters at spring tide. Depending on turbulent characteristics and wave-current interactions, some suspended sediments formed flocks and settled in lower hydrodynamic energy zones within the sheltered area, while others were transported back to the sea. Wave overtopping and wave breakdown above the low-crested breakwaters caused the water level to rise, piling up and generating strong backflows around the gap. The wave breaking on the submerged breakwaters altered the longshore current, causing the longshore sediment drift to settle behind them, creating a new shoreline (Ratnayake et al., 2018). Munari et al. (2011) presented a similar study, in which a semi-submerged breakwater changed the alongshore sediment transport at Punta Marina, north-eastern Italy. Sulaiman and Hidayat (2020) found that low-crested structures created a rotary water current pattern, slowing down the longshore current velocity and causing rapid sediment deposition behind the submerged breakwater. The breakwater acted as a sedimentary trap, allowing the external water current to carry the sediment through the gaps during high tide and flow out during low tide. On the other hand, submerged breakwater impacts on hydrodynamics can create undesired consequences. Gallerano et al. (2020) and Vona et al. (2020) reported that submerged breakwaters were an obstacle to sediment transport, negatively affecting nourishment processes. Zanuttigh (2007) showed that erosion around low-crested structures was linked to a flux of wave overtopping. Rip currents at gaps created a flame-shaped erosion while inducing a crescent-shaped erosion at the roundheads.

### 2.4 Impact on ecology

Submerged breakwaters also play imperative roles in coastal ecology and nearshore environments by providing unnatural sheltered habitats. A case study by Stender et al. (2021) clearly depicted that submerged breakwaters provided an exemplary area for coral to flourish while protecting the Kahului Commercial Harbor from large ocean swells. Burt et al. (2009) conducted a study in Dubai and discovered that submerged breakwaters acted as large-scale man-made reefs that sustained a wide range of marine communities, offering greater hard-bottom habitats than traditional artificial reefs. They also found that construction materials used to build the breakwaters could promote coral recruitment. They also suggested that gabbro was more preferable and workable compared to concrete and sandstone.

Acting as artificial habitats for marine species, submerged breakwaters are known to have noticeable impacts on marine biodiversity. A pilot study carried out at Kovalam, India, by Kumar et al. (2014), indicated that epibiotic assemblages were grown on submerged breakwaters. In Italy, Bertasi et al. (2007) also found an increased microbenthic species richness at low-crested breakwater. The biotic assemblage might reflect that the low-crested coastal protection structure was eco-friendly. A similar study by Moschell et al. (2005) concluded that submerged breakwaters were like natural rocky coasts in terms of their ecological roles, which influenced colonizing marine epibiota. They also could alter the distribution of hard-substrate species and propagate invasive species, affecting the identity of native benthic communities. Since submerged breakwaters have relatively more underwater surface area, they allow more species to settle and survive over time, increasing diversity and biomass. Moschell et al. (2005) also concluded that submerged breakwaters might alter the abundance and composition of epibiotic species, in turn controlling algae growth and enhancing species diversity for recreational activities. The habitat values of two submerged breakwaters in Mobile Bay, USA, were assessed by Scyphers et al. (2014), who found that these breakwaters were feasible and offered habitats for mobile invertebrates, filter-feeding bivalves, and fish populations. Munari et al. (2011) and Munari (2013) studied the impact of an offshore semi-submerged breakwater on benthic community functional trait patterns and invertebrate assemblages at Punta Marina, Italy. They showed that the taxonomic composition of the benthic population at the landward and seaward zones of the semi-submerged breakwater was varied. They also found an increase in macroalgae and associated amphipods on the leeward side of the breakwater, remarking that the environmental stability created at the leeside of the breakwaters allowed a more complex benthic community to develop.

### 2.5 Impact on coastal tourism and recreation

Submerged breakwaters can be utilized for tourism and recreational purposes. There seems to be unanimous agreement that submerged breakwaters can sustain the tourism industry within a coastal community while still offering adequate beach protection (Kuriyama and Banno, 2018; Nyoman et al., 2019; Vu et al., 2019). Coastal areas with submerged breakwaters can be attractive tourism destinations, since beach aesthetics are not interrupted. Ranasinghe and Turner (2006) claimed that submerged breakwaters did not cause any beach amenity loss or negative aesthetic influences. Zahra (2018) highlighted that submerged breakwaters neither alter beaches nor block sight of horizons. Pradjoko et al. (2015) further evaluated submerged breakwaters and suggested that they were appropriate for coastal protection at Gili Trawangan, Lombok, Indonesia, due to their aesthetics and environmental considerations. The study by Pranzini et al. (2018) stated that placing submerged breakwaters further offshore could create more recreational spaces, as well as prevent any hazards linked with beachgoers and the structures. Concessionaires associated with the increased beach width could increase income.

### 2.6 Others impacts

Submerged breakwaters pose other possible environmental impacts in both the short- and long-term. A few studies related to the impacts of submerged breakwaters on navigational activities have been published. Submerged breakwaters might be serious invisible hazards to boats and swimmers (Masria et al., 2015; Van Rijn, 2011). Patnaik and Kumar (2015) stated that submerged breakwaters were difficult to construct in marine environments and could induce navigation risks.

## 3 Emerged breakwaters

Emerged breakwaters are coastal structures with their crests above a designed water level to limit wave overtopping. They have been widely adopted for harbors and coastal protection (Uda, 2022). Emerged detached rubble mound breakwaters are a prevalent type of coastal protection structures in the United States of America (Hardaway and Gunn, 2010), Europe (Anfuso et al., 2011; Araújo et al., 2014; Armaroli et al., 2009; Dolphin et al., 2012), and Japan (Sane et al., 2007; Uda, 2016). Different construction materials used to build them include natural rocks, concrete units, and geotextiles (Saengsupavanich 2013a, 2013b). Many experimental and theoretical studies have been undertaken to investigate their efficiency, but such a topic is not within the scope of this review. On the other hand, our article is interested in the fact that emerged breakwaters induce many types of positive and negative environmental impacts, generated during their pre- and post-constructions. In this section, the environmental impacts of emerged breakwaters on coastal environments are well-compiled and summarized under different sub-categories.

### 3.1 Economic considerations

Emergent breakwaters have relatively higher construction costs compared to other soft coastal protection options. Their design is not a straightforward process but is an iterative technique that includes an initial design phase based on mathematical or physical modelling, design testing, and fine tuning, such as geometric design of the breakwater cross-section (Capobianco et al., 2002). In Thailand, the construction cost of emerged detached breakwaters located approximately 50 m from the shoreline was approximately 1.9 million USD per 1 km of coastline (Saengsupavanich, 2013a). The construction budget could greatly vary, depending on domestic labor and material prices (Hillen et al., 2010).

Emerged breakwaters provide an effective defense mechanism to eroding coasts. From the economic viewpoint, damages averted from the construction of breakwaters were considered benefits (Males and Melby, 2011). In Malaysia, a large amount of sediment was accumulated on beaches in a short period of time, illustrating the effectiveness of emerged breakwaters in increasing beach elevation (Mohamed Rashidi et al., 2021) and implying a positive economic impact, because more land area was acquired. In Thailand, once-eroded shoreline became stabilized by offshore emerged breakwaters, increasing the community’s confidences to invest, developing the coastal area, and promoting local economy (Saengsupavanich et al., 2009). Another possible secondary economic benefit received from emerged breakwaters was wave power generated by breakwater-mounted instruments (Contestabile et al., 2016; Mustapa et al., 2017).

### 3.2 Impact on beach morphology

It has long been realized that emerged breakwaters significantly induce shoreline morphological changes in the surrounding area after their installation. Lorenzoni et al. (2016) concluded that, depending on the breakwater configuration, beaches were totally changed. Emerged breakwaters produced lower and narrower berms. Pranzini et al. (2018) found that swash motion caused immediate morphological changes associated with an emerged berm, which highly depended on the breakwater dimensions. Frihy et al. (2004) discovered that the breakwaters at the Baltim and the Ras El Bar beaches in Egypt affected the grain size distribution of beach and surficial sediments. The beach behind the detached breakwaters gradually coarsened landwards. This pattern was caused by erosion and accretion actions from grain sorting processes. Another study by Saengsupavanich (2013b) revealed that the detached emerged breakwaters on a muddy coast in Thailand increasingly induced sedimentation on the leeward side of the breakwaters after the construction was completed. It took two years for the mud to become dense and thick.

Tombolos and salients are produced by emerged breakwaters. The effectiveness of emerged breakwaters and the formation of tombolos or salients, are dependent on relationships amongst the shoreline-breakwater distance, the breakwater’s length, and the gap width (Ramanujam and Sudarsan, 2003; Razak and Nor, 2018; Saidi et al., 2012a). Saidi et al. (2012b) undertook a study along the coast of Hamman-Lif, Tunisia, and concluded that the breakwaters which were the longest, closest to the shoreline, and less spaced, could form well-developed tombolos. Alternatively, the emerged breakwaters which were short, located far from the coastline, and far from each other caused very small tombolos and even salients. Saengsupavanich (2013a) found that people living along the Nakhon Si Thammarat coastline, Thailand, preferred the tombolos, since local communities could relax and utilize the widened protected beach. The curving shoreline resulted from the detached breakwaters was insignificant, compared to the losses of property and life due to wave attacks (Saengsupavanich et al., 2009).

Updrift deposition and downdrift erosion are other consequences after installing emerged breakwaters. A study by Saidi et al. (2012a) provided evidence of beach response to the emerged breakwater construction. A single breakwater at Redes, Tunisia, and two successive detached breakwaters at Ezzahra created embayments (salients and tombolos), updrift deposition, and downdrift erosion. Frihy and Deabes (2012) reported that downdrift erosion was evident at El Alamein Resorts on the western Mediterranean coast of Egypt. Many previous publications presented the same findings, that the emerged breakwaters intercepted alongshore sediment transport, inducing downdrift erosion (Dolphin et al., 2012; Pranzini et al., 2018). The magnitude and patterns of accretion and erosion resulted from waves breaking at large oblique angles to the shoreline. Dolphin et al. (2012) who analyzed the influence of nine breakwaters at Sea Palling, North Sea, found that downdrift shoreline began to be eroded in response to reduced sediment supply from the updrift direction. Frihy et al. (2004) concluded that deposited sediment between each emerged breakwater created bulges of tombolo, changing the breakwater system into a shore-parallel seawall, totally blocking sediment flow behind the lee of the breakwaters, worsening the downdrift erosion.

### 3.3 Impact on hydrodynamics

Emerged breakwaters create complex hydrodynamic characteristics in terms of wave height, water flow, and sediment movement. Gaps between the emerged breakwaters and their orientations influence wave energy dampening (Jackson et al., 2015). According to Kamali et al. (2010), narrower gaps between detached emerged breakwaters were more efficient in lowering wave energy, which could protect eroding beaches with minimal consequences than other hard structures. The analysis carried out by Ilic et al. (2005) confirmed that wave transmission, shoaling, diffraction, refraction, wave-current interaction, and non-linear interaction all contributed to wave transformations around emerged breakwaters in shallow water regions. Lorenzoni et al. (2016), who compared efficiency between emerged and the submerged breakwaters, concluded that emerged breakwaters were more effective than submerged ones because of the fact that the former could restrict both wave transmission and water piling-up in sheltered areas, reducing sediment movement within swash zones.

Differences in hydrodynamics characteristics in front of, behind, and between gaps of emerged breakwaters have been observed by many researchers. Masucci et al. (2019), who applied plaster balls in tetrapod breakwaters on Okinawa Island, Japan, showed that the plaster balls in front of the emerged breakwaters became smaller than those installed at the lee of the breakwaters. The wave energy in front of the breakwaters was higher because of wave reflection and breaking against a breakwater slope. Frihy et al. (2004) discovered that the detached emerged breakwaters at Baltim beach, Egypt, induced salient and tombolo formations, confining water current in the leeside of the breakwaters, generating serious eddies with a very high velocity. A zone with reduced wave energy behind the breakwaters or a rip current between the breakwaters’ gap could affect sea bathing and tourism activities (Ferrari et al., 2019). Archetti and Zanuttigh (2010), who monitored the hydro-morphodynamic changes of a beach protected by detached breakwaters, found deep scouring between the breakwaters’ gaps, which resulted from the rip current. Similarly, Archetti et al. (2012) attempted to adjust breakwater layouts in order to decrease the strong currents occurring between the gaps and the roundheads of breakwaters.

### 3.4 Impact on ecology

Emerged breakwaters can have different impacts on ecology, depending on the environmental setting where they are built. Fish and benthic assemblages can be affected in terms of diversity, abundance, and ecological state (Burt et al., 2011; Hammond et al., 2020; Mamo et al., 2021). Colosio et al. (2007) highlighted that breakwaters provided artificially protected conditions that improved fine sediment deposition and attracted non-native marine species. Diel variation in the feeding habits of juvenile catfish around offshore breakwaters was studied by Yamazaki et al. (2019), who found that catfish juveniles were more abundant in the evening and night around offshore breakwaters, indicating that they had moved out the breakwater shelter after sunset, and the breakwaters might reduce the risk of predation from other piscivore fish. In contrast, Becchi et al. (2014), who analyzed the ecological effects of breakwater systems on soft-bottom assemblages along the North Tyrrhenian coast, found that breakwater impact was limited to only a small, restricted area. Anton et al. (2019) conceptually assessed the impacts of coastal protection structures on Black Sea biocenosis and found that emerged breakwaters could catastrophically impact zoobenthos due to the direct mechanical destruction of habitats and benthic populations. They also mentioned that breakwaters severely affected phytoplankton by reducing the amount of light and sediment resuspension, decreasing the concentration of dissolved oxygen. Bacchiocchi and Airoldi (2003) concluded from their study that breakwaters might change the distribution of locally abundant species rather than increase species variety.

Coral communities can be affected by the presence of emerged breakwaters. Masucci et al. (2019) measured water depth, sediment characteristics, wave energy, coral cover, and the benthic community around tetrapod breakwaters at Ogimi Village, Japan, and found the interesting result that living hermatypic corals were almost completely absent in front of and behind the tetrapod breakwaters. Although the breakwaters caused sedimentation behind their lees, the relatively flat areas around them might not be optimal for coral larvae settlement. The shallow area at the lee of the breakwaters could further impact the coral communities by increasing ultraviolet exposure. Moreover, the sedimentation, heavily loaded with organic matters, and its plume could intensify turbidity and bacterial activity, worsening coral diseases and coral survival rates. Similar findings were obtained by Burt et al. (2010), who showed that the lee side of breakwaters exhibited poor coral cover with high coral mortality and suggested that the leeward zone was improper for coral community development.

There have been a few studies on the supportive role of emerged breakwaters in promoting mangrove progradation. Kamali et al. (2010) studied the intertidal muddy beach in Selangor, Malaysia, where emerged breakwaters were used for a mangrove restoration scheme. The segmented breakwaters allowed water circulation and avoided negative ecological consequences. The breakwaters provided a calm environment, facilitating mangrove recovery without replanting. Similarly, the breakwaters built at Karimunting and Penibung Bay, Indonesia, promoted mangrove rehabilitation, which was evident from the high colonization rate of Avicennia marina and Rhizophora sp. (Akbar et al., 2017).

Algal and seagrass ecosystem are influenced by emerged breakwaters. Martins et al. (2009) found that emerged breakwaters could alter local algae ecosystem. The effects of a reduction in hydrodynamics included a replacement of barnacles, limpets, and frondose algae by an increasing cover of ephemeral algae, implying that the artificial sheltering of naturally exposed coasts could promote a shift from consumer-to producer-dominated communities.

Bacchiocchi and Airoldi (2003) revealed that epibenthic assemblages, such as mussels and green ephemeral algae, quickly colonized breakwaters. A case study by Carugati et al. (2018), who investigated the impact of breakwater relocation, found that sediment features were altered, and seagrass meadows had doubled in total organic matter.

Certain marine species, such as sea urchins, are affected by breakwaters (Bauman et al., 2016; Burt et al., 2011; Yu, 1998; Scheibling and Raymond, 1990). Sea urchins are important herbivores on coral reefs, since they play an important role in maintaining the coral-algae balance. The embryogenesis of the sea urchin is a suitable bioindicator of seawater and sedimentation quality in impacted ecosystems (Lukyanova et al., 2017). The presence of sea urchins can significantly influence breakwaters and the dynamics of reef benthic communities by enhancing topographic complexity and minimizing algae and sediment settlement (McClanahan and Muthiga, 2013). In Dubai, Bauman et al. (2016) concluded that sea urchin availability was shown to be lowest at the leeward side of breakwaters.

### 3.5 Impact on coastal tourism and recreation

Emerged breakwaters bring a positive impact to the coastal tourism and recreation sectors. Jackson et al. (2015) highlighted that detached emerged breakwaters could improve the recreational amenity of a beach by providing positive and enjoyable benefits. El-Masry (2022) reported that dolos emerged detached breakwaters were implemented in Alexandria city, Egypt, to provide a safe and secure area for swimming activities. Saengsupavanich (2013b) reported that detached breakwaters in Thailand could protect the coastline while promoting tourism and supporting local activities and relaxation. Another study in Thailand showed that public rest huts were constructed to promote eco-tourism along the breakwaters on a muddy coastline. When the coastline was protected, local communities felt secure, and further livelihood development could follow Saengsupavanich (2013a).

On the other hand, some publications have mentioned that emerged breakwaters generate negative disturbances, such as deteriorated sea landscapes and beach utilization (Lamberti and Zanuttigh, 2005). Cappietti (2011) claimed that emergent breakwaters made seascapes less natural, while stating that such impacts could be reduced by lowering crest height and widening crest width to maintain the same transmission coefficient. Frihy et al. (2004) reported that detached breakwaters could obstruct swimming activities in summer, because strong water currents and eddies were produced between gaps of breakwaters, increasing the potential for drowning. The number of drowning accidents tended to substantially increase each summer, with an average of 67 victims/year.

### 3.6 Others impacts

The literature has suggested that seawater quality can be affected by emerged breakwaters both positively and negatively. Lamberti et al. (2005) mentioned that active and complex current circulations presenting around breakwaters create an intense mixing of the water, causing a positive effect for the water quality. The questionnaire survey in Lamberti et al. (2005) showed that the respondents preferred emerged breakwaters in terms of water quality and being child-friendly. On the contrary, Elsharnouby et al. (2012) highlighted that the installation of emerged breakwaters had an adverse impact on the water quality, because of the rapid deterioration of the seawater within the protected area. In addition, the study by Carugati et al. (2018) reported that the breakwaters along the coastline of Gabicce Mare altered the current circulation and had a significant impact on water quality. Improper breakwater design led to hypoxia and reduced water quality in the coastal areas. The breakwaters created water stagnation, resulting in hypoxic conditions in the summer, poor water quality, and low beachgoer satisfaction. However, these issues were resolved by relocating the breakwaters. Poor water quality caused by breakwaters had been mentioned by the previous work of Yu (1998), who experimented with the water quality around breakwaters in Korea.

## 4 The way forwards to sustainably managing coasts with breakwaters

Breakwaters, both submerged and emerged, have been implemented in coastal areas, bringing with them various environmental impacts, depending on their locations, including coastal morphology, hydrodynamics, ecology, and tourism and recreation (Figure 1). Their impacts may vary when combined with other coastal protection works (Rahmawati et al., 2021; Schoonees et al., 2019). Although it cannot be denied that breakwaters perform their functions well in dissipating waves, many researchers have pointed out that they may work little with nature, and sustainability is currently a critical issue (Gracia et al., 2018). Despite the fact that much research has been conducted to better understand the behaviors and processes involved with breakwaters, there are still a lot of unknown questions regarding their environmental impacts.

**Figure 1:** Environmental impact of submerged and emerged breakwaters.

What seem to be clear are breakwater impacts on beach morphology and hydrodynamics. Conclusions about such physical impacts (such as wave dissipation effectiveness, updrift accretion, downdrift erosion, the formation of tombolo or salient, flanking, scouring, eddies, and rip currents) are in the same direction. The most noticeable impact, that can be visually realized, is updrift deposition and downdrift erosion, that happen for both submerged and emerged breakwaters. In some cases, submerged breakwaters induce neighboring shoreline erosion at both updrift and downdrift sides simultaneously, due to flanking phenomenon (Torres-Freyermuth et al., 2019). Knowledge on salient and tombolo formations, depending on relationships amongst the shoreline-breakwater distance, the breakwater’s length, and the gap width, are well-established for emerged breakwaters (Ramanujam and Sudarsan, 2003; Razak and Nor, 2018), but seems underdeveloped for submerged ones (Kubowicz-Grajewska, 2015). Leeward sedimentation is enhanced by submerged breakwaters. While creating a rotary water current pattern, wave overtopping on submerged breakwaters induces a suspended sediment flow on the leeward side, slowing down the longshore current velocity, resulting rapid sediment deposition behind them (Fitri et al., 2019; Sulaiman and Hidayat, 2020). The characteristics of dynamics and processes that drive shoreline responses are basically different for submerged and emerged breakwaters (Tunji et al., 2012). Submerged and emerged breakwaters have been negatively criticized for their rip current effects (Chang et al., 2018; Frihy et al., 2004; Liu and Wu, 2022; Yin et al., 2018). Although gaps between emerged breakwaters are necessary for constant water exchange, they induce tombolos, rip currents, scouring, and bed irregularities (Frihy et al., 2004; Jackson et al., 2015; Razak and Nor, 2018; Saidi et al., 2012a). These physical impacts are what the eyes can see and have been extensively studied, both in the field and in laboratories. After reading Section 2.2, Section 2.3, Section 3.2, and Section 3.3 of this article, coastal practitioners can make unambiguous decisions on how to manage breakwater impacts on beach morphology and hydrodynamics.

Conversely, what seem to be unclear are breakwater impacts on ecology. It is clear that both emerged and submerged breakwaters destroy benthic communities during their construction (Anton et al., 2019), but alter marine species community in a longer term (Scyphers et al., 2014). Although many researchers have shown that breakwaters alter pristine ecology, none of them cannot conclude whether such changes are positive or negative. For example, breakwaters can increase epibiotic assemblages and microbenthic species richness, which in turn, control algae growth (Bertasi et al., 2007; Kumar et al., 2014). How do we decide whether to preserve algae or to promote macrobenthos? Another example is based on the fact that breakwaters increase marine biodiversity (Hammond et al., 2020; Mamo et al., 2021), yet how can we be certain that increased biodiversity is good for the original ecological food web? Martins et al. (2009) found that breakwaters generated the replacement of barnacles and limpets by an increasing cover of ephemeral algae, accelerating a shift from consumer-to producer-dominated communities. Is changing to producer-dominated biocenosis good or bad? Additionally, the ecological impacts of breakwaters may be location-specific to and dependent on the existing marine environment at such a site. Results obtained from a study in a tropical country may be different from those of a high-latitude country. For instance, a country with or without sea urchins may exhibit a different result concerning the algal community around breakwaters, as supported by McClanahan and Muthiga, (2013) who showed that the presence of sea urchins affected algae growth. Therefore, it can be implied that the current status of the research on breakwater impacts on ecology is still far from completion.

Regarding tourism and recreation, there is a unanimous agreement that submerged breakwaters do not destroy beach aesthetics and promote tourism (Pradjoko et al., 2015; Pranzini et al., 2018). However, for emerged breakwaters, there are many disagreements about their impacts on the tourism, depending on how researchers want to persuade readers. Since beach beauty is a personal preference, no researcher is in a proper position to judge whether emerged breakwaters promote or demote it. Criticizing whether emerged breakwaters enhance or deteriorate coastal community livelihoods or the surrounding environment is subjective and is totally based on the researchers’ judgments. Some researchers advocate for emerged breakwaters, while some publications demote them. Jackson et al. (2015) and Saengsupavanich et al. (2013a) concluded that breakwaters supported tourism and recreational activities, while Lamberti and Zanuttigh (2005) claimed that breakwaters reduced beach utilization. Another example is the discrepancy in the impact on water quality surrounding breakwaters. While Lamberti et al. (2005) argued that breakwaters created a positive effect on water quality by intense mixing, Elsharnouby et al. (2012) claimed that breakwaters had a significant impact on water quality and induce hypoxia (Carugati et al., 2018). Coastal managers need to be careful when deciding whether breakwaters are good or bad. A coin always has two faces.

Future developments on ecology-friendly breakwaters are needed. It is undeniable that breakwaters are still necessary in certain situations, but how they can support coastal development while promoting environmental conservation is still challenging. Bridging the gap between coastal structures and nature conservation is vital, as they provide benefit and support greater environmental good (Jordan and Fröhle, 2022). Designing coastal structures is not difficult since there are many formula and guidelines readily available (Saengsupavanich, 2017; Saengsupavanich and Pranzini, 2022), but how to enhance environmental conditions at the same time is not easy. Recent attempts have been conducted by many researchers to increase ecological functions of breakwaters. Ostalé-Valriberas et al. (2018) created tidepools, which are unique intertidal habitats that favor breeding and feeding as well as providing shelter to a certain group of species, on artificial substrates in an attempt to mitigate the negative effects of artificial substrates on marine biodiversity. Kim et al. (2020) combined a submerged breakwater with an artificial reef installation to compensate for the stability problem caused by local scour. The artificial reefs are also known to increase marine biodiversity, thus a have great potential to stabilize the breakwaters while promoting the environment (Nguyen et al., 2022). To be more nature-friendly, submerged reefs constructed from recycled mollusk shell were introduced by Corbau et al. (2022). Meanwhile, oyster reef breakwaters as well as oyster towers with recruited oysters, acting as emerged breakwaters, have also been shown to damp waves while trapping sediment (Chowdhury et al., 2021). Additionally, research on modifying an armor layer of breakwater has been recently conducted in a hope to enhance its wave-dissipating effectiveness and ecological functions. MacArthur et al., (2020) showed that a suitable rock selection and a deliberate placement of armor rocks could increase the availability of limpets. Almaghraby et al. (2022) tested hollow artificial shells mounted on rubble mound breakwater, in order to use shapes from nature to dissipate waves. It was found that the partially submerged shell-mounted breakwaters had better efficiency, particularly in areas with short coastal waves, and the crest width of the submerged breakwater could be reduced less than half, by deploying the artificial shell. Coastal researchers must continue to search for breakwaters that are both effective in battling waves and in being able to enhance the environment.

## 5 Conclusion

Managing the environmental impacts of breakwaters is a significant and burgeoning challenge for coastal stakeholders. Submerged and emerged breakwaters have been widely implemented worldwide, yet they have been found to induce many undesirable environmental consequences. In this review article, economic consideration and impacts on beach morphology, hydrodynamics, ecology, and beach utilization are summarized in order to help coastal practitioners sustainably manage coastlines with breakwaters while also lessening environmental disturbances. Since the current knowledge about breakwater impacts is still limited, and conclusions made by different researchers are sometimes in disagreement, coastal decision makers should thoroughly consider every environmental aspect to ensure safe and sustainable coastline.

## Declarations

### Author contribution statement

All authors listed have significantly contributed to the development and the writing of this article.

### Funding statement

This research did not receive any specific grant from funding agencies in the public, commercial, or not-for-profit sectors.

### Data availability statement

Data will be made available on request.

### Declaration of interest’s statement

The authors declare no competing interests.

### Additional information

No additional information is available for this paper.
